The article "Study on Mechanism of Jiawei Chaiqin Wendan Decoction in Treatment of Vestibular Migraine Based on Network Pharmacology and Molecular Docking Technology" was published in 2021. Journal: Evid Based Complement Alternat Med.

# Study on Mechanism of Jiawei Chaiqin Wendan Decoction in Treatment of Vestibular Migraine Based on Network Pharmacology and Molecular Docking Technology

**DOI:** 10.1155/2021/5528403

**Published:** 2021-10-31

**Authors:** Menglin Liu, Genhao Fan, Daopei Zhang, Mingjun Zhu, Huailiang Zhang

**Affiliations:** ^1^Henan University of Traditional Chinese Medicine, Zhengzhou 450000, China; ^2^Tianjin University of Traditional Chinese Medicine, Tianjin 301617, China; ^3^The First Affiliated Hospital of Henan University of Chinese Medicine, Zhengzhou 450000, China

## Abstract

**Objective:**

To predict the main active ingredients, potential targets, and key pathways of Jiawei Chaiqin Wendan decoction treatment in vestibular migraine and explore possible mechanisms by network pharmacology and molecular docking technology.

**Methods:**

The active ingredients and related targets of Jiawei Chaiqin Wendan decoction were obtained from the Traditional Chinese Medicine Systems Pharmacology Database and Analysis Platform (TCMSP). The corresponding genes of the target were queried by UniProt database, and the “drug-compound-target-disease” network was constructed by Cytoscape 3.7.2 software. GO functional enrichment analysis and KEGG pathway enrichment analysis were carried out by R software and Bioconductor, and column chart and bubble chart were drawn by Prism software and OmicShare database for visualization. Finally, the mechanism and potential targets of Jiawei Chaiqin Wendan decoction in the treatment of vestibular migraine were predicted.

**Results:**

The “drug-compound-target-disease” network contains 154 active ingredients and 85 intersection targets. The key targets include AKT1, IL6, MAPK3, VEGFA, EGFR, CASP3, EGF, MAPK1, PTGS2, and ESR1. A total of 1939 items were obtained by GO functional enrichment analysis (*P* < 0.05). KEGG pathway enrichment analysis screened 156 signal pathways (*P* < 0.05), involving PI3K-Akt signal pathway, AGE-RAGE signal pathway in diabetes complications, MAPK signal pathway, HIF-1 signal pathway, IL-17 signal pathway, etc. Molecular docking results showed that quercetin, luteolin, kaempferol, tanshinone IIa, wogonin, naringenin, nobiletin, dihydrotanshinlactone, beta-sitosterol, and salviolone have good affinity with core target proteins IL6, PTGS2, MAPK1, MAPK3, and CGRP1.

**Conclusion:**

The active ingredients in Jiawei Chaiqin Wendan decoction may regulate the levels of inflammatory factors and neurotransmitters by acting on multiple targets such as IL6, MAPK3, MAPK1, and PTGS2, so as to play a therapeutic role in vestibular migraine.

## 1. Introduction

Vestibular migraine (VM) is a chronic and disabling disease that is common and has a genetic tendency; the main symptoms are recurrent dizziness/vertigo, which may be accompanied by nausea and vomiting with or without headache [1]. Studies have shown that VM is one of the common causes of recurrent dizziness or vertigo [1,2]. VM can occur at any age, and the ratio of male to female is 1 : 1.5–1 : 5, and it is more common in women [3]. VM is generally regarded as a subtype of migraine. Since a new hypothesis was published in the Lancet in 1979, it has been proposed that trigeminal neurovascular system containing neuropeptides plays an indispensable role in migraine. Up to now, trigeminal neurovascular system has been widely regarded as the basis of this highly complex nervous system disease for 40 years [4]. At present, the pathogenesis of VM is still not completely clear at home and abroad, and the basis of pathogenesis may be associated with ion channel defect and cortical spreading depression (CSD). CSD activates the trigeminal neurovascular system, and the trigeminal ganglion releases calcitonin gene-related peptides (CGRP), substance P, and other neuropeptides, causing meningeal vascular inflammation, and thus leading to migraine symptoms. In addition, the overlap of the pathways responsible for pain and balance in the central nervous system, the fibrous connection between the trigeminal nucleus and the vestibular nucleus, and the trigeminal nerve innervating the inner ear eventually lead to vestibular symptoms [5].

The diagnosis of VM is mainly based on the characteristics of the patient's clinical onset and lacks specific signs and objective diagnostic basis. In the past few decades, uncertainty about the diagnosis of VM has limited the progress of treatment [6]. There is insufficient evidence to support the use of drugs for VM treatment. Sometimes, western drugs are effective in preventing migraine, but their role in VM treatment is not clear, and the effect of these drugs on VM prevention cannot be verified [7]. Recurrent dizziness or vertigo has a significant impact on patients' quality of life and their psychology. Extensive examinations and long-term treatment impose a huge economic burden on patients' families and society. It is obvious that further research on potential new treatments for VM therapy is needed. Vestibular migraine is characterized by dizziness or vertigo, visual rotation, instability, and current or previous migraine, which can be classified as “xuan yun” in traditional Chinese medicine. The earliest description of “xuan yun” in traditional Chinese medicine can be mentioned in the “Canon of Medicine.” Doctors of various dynasties had different understandings of “xuan yun,” with different emphasis on syndrome differentiation and treatment. And to sum up, there are five aspects: wind, fire, phlegm, deficiency, and blood stasis. In the treatment of vertigo, traditional Chinese medicine has unique advantages. A study has compared the curative effect of TCM syndrome differentiation treatment and conventional western medicine treatment on patients with vertigo and found that, compared with conventional western medicine treatment, TCM syndrome differentiation treatment of vertigo can more effectively improve the clinical symptoms of patients [8].

Chaiqin Wendan decoction is made of Wendan decoction from Yao Sengyuan in the Southern and Northern dynasties. The modified Chaiqin Wendan decoction (JCWD) is an effective empirical prescription for the treatment of vertigo in clinic. This prescription is composed of Radix Bupleuri (Chaihu), Radix Scutellariae (Huangqin), Pinellia tuber (Banxia), Dried tangerine Peel (Chenpi), Fructus Aurantii Immaturus (Zhishi), Poria cocos (Fuling), Radix Paeoniae Alba (Baishao), Angelica sinensis (Danggui), Salvia miltiorrhiza (Danshen), Gastrodia elata (Tianma), Uncariae Ramulus Cumuncis (Gouteng), and Shi Cassia (Shijueming). At present, clinical observation indicates that Chaiqin Wendan decoction has a significant effect on the treatment of patients with dizziness and headache caused by Triple Burner Congestion [9–11]. There have been some studies based on network pharmacology to reveal the molecular mechanism of TCM treatment of diseases. This study aims to predict the potential target and mechanism of JCWD in treating VM through network pharmacology and molecular docking methods.

## 2. Materials and Method

### 2.1. Acquisition of Active Ingredients and Targets of TCM

The TCMSP (http://tcmspw.com/tcmsp.php) [12] database was used to search the TCM in JCWD formulae (Radix Bupleuri, Radix Scutellariae, Pinellia tuber, Dried tangerine Peel, Fructus Aurantii Immaturus, Poria cocos, Radix Paeoniae Alba, Angelica sinensis, Salvia miltiorrhiza, Gastrodia elata, Uncariae Ramulus Cumuncis, and Shi Cassia), with two parameters related to ADME (absorption, distribution, metabolism, and excretion), namely, oral bioavailability (OB greater than or equal to 30%) and class medicinal (DL greater than or equal to 0.18) for screening of TCM active ingredients. Based on TCMSP and DrugBank databases, the targets of active ingredients were retrieved by Perl software and UniProt KB (http://www.uniprot.org/), and gene annotation was performed.

### 2.2. Obtain the Intersection Genes of TCM and Diseases

Using GeneCards (https://www.genecards.org/) and OMIM database (https://omim.org/) by retrieving “vestibular migraine” look up vestibular migraine related genes and remove duplicates. Through Venny2.1 software, the target of active ingredients of traditional Chinese medicine obtained above was intersected with disease-related genes.

### 2.3. Draw “Drug-Compound-Target” Network

The information of drug name, drug active ingredient, gene target of intersection between drug and disease, and the relationship network among them were imported into Cytoscape3.7.2 software to construct the network diagram of “drug-compound-target” for visual analysis.

### 2.4. Protein-Protein interaction (PPI) Network and Core Gene Network

Multiple proteins were introduced into String11.0 (https://string-db.org/), and the species was selected as “*Homo sapiens*,” with a medium confidence of 0.400 to predict the associated PPI network. Download protein-protein interaction TSV file, import Cytoscape3.7.2 software, and use CytoHubba plug-in to screen core target proteins.

### 2.5. GO and KEGG Enrichment Analysis

There is the core target gene ID through the R software and Bioconductor (http://www.bioconductor.org) to GO functional annotations and KEGG pathway enrichment analysis. *P* < 0.05 was selected for functional annotation clustering. In order to study the biological effects of VM targets of drug therapy by regulating specific pathways, the top 10 items were screened according to the enrichment degree and a bar chart was drawn. Similarly, *P* < 0.05 was selected as the significant pathway for cluster analysis, and the top 20 items were screened according to the enrichment degree to draw a bubble plot.

### 2.6. Molecular Docking

The 2D structures of key compounds were downloaded in PubMed (https://www.ncbi.nlm.nih.gov/pubmed). The 3D structures of ligands were generated by Chem3D software, and their energy was minimized and exported to mol2 format. All compounds were saved as ligand parameter files in pdbqt format by AutodockTools-1.5.6 software. The 3D structure of the core target protein was downloaded from PDB database (https://www.rcsb.org/) and saved in PDB format. The solvent and water molecules in the target protein receptor molecules were removed by pymol software. Then, the protein receptor molecules were hydrogenated and calculated by AutodockTools software and saved in pdbqt format. After the ligand and protein receptor molecular preprocessing is completed, the appropriate box center and box lattice parameters are set by AutodockTools-1.5.6 software, the active pocket sites that small molecular ligands may bind to are included, and the parameter text file is set, and the other parameters remain default. Molecular docking was carried out by Autodock Vina, and 3D diagrams were drawn by PyMol software for the docking results with the strongest binding activity of each target protein to show the hydrogen bond and hydrophobic effect formed by it.

## 3. Results

### 3.1. Collection of Active Components and Targets of JCWD

A total of 221 active components of TCM, which were OB ≥ 30% and DL ≥ 0.18 in JCWD formulae, were retrieved by TCMSP database. The basic information of some active components of JCWD is shown in Table 1. Based on TCMSP and DrugBank database, a total of 3376 protein targets related to the above active ingredients were obtained by Perl software, and 1531 gene symbols were obtained after gene annotation using UniProt KB.

### 3.2. Intersection Targets of JCWD and VM

In GeneCards (https://www.genecards.org/) and OMIM database (https://omim.org/) by retrieving “vestibular migraine” search related genes, a total of 826 were extracted after duplication. Through Venny2.1 software, the intersection of traditional Chinese medicine target and disease genes was obtained, and 85 genes related to JCWD treatment of VM were obtained, as shown in Figure 1.

### 3.3. Construction of “Drug-Ingredient-Target” Network

First, the intersection between drug targets and disease genes is obtained, and then the information such as VM related genes, active ingredient targets of traditional Chinese medicine, and their interrelation network are imported into Cytoscape3.7.2 software for visual analysis, and the “drug-active ingredient-target” network diagram is constructed. The network consists of 249 nodes (10 TCM name nodes, 154active ingredient nodes, and 85 gene target nodes) and 915 edges, as shown in Figure 2. The average degree value of this network is 7.66, and the top 10 active ingredients were screened according to the degree value, as shown in Table 2, among which the degree values of quercetin, luteolin, kaempferol, tanshinone IIa, and wogonin are greater than or equal to 16 (more than 2 times the average value). In addition, quercetin, luteolin, kaempferol, naringenin, nobiletin, and *β*-sitosterol are the common active components in many TCMin JCWD, which can interact with 53, 21, 19, 13, 13, and 12 target proteins, respectively. The top 10 target genes in screening value were PTGS2, HSP90AA1, SCN5A, AR, ADRB2, ACHE, ESR1, NOS2, PPARG, and GABRA1, which could interact with 136, 91, 84, 70,62, 53, 43, 41, 35, and 28 active components, respectively.

### 3.4. Protein-Protein Interaction Network (PPI) and Core Gene Network Were Constructed

Eighty-five JCWD gene targets for VM treatment were introduced into String11.0 to construct a Protein-protein interaction network (PPI), and isolated nodes were removed, as shown in Figure 3. Then, the top 20 key genes were screened out according to the Degree value, as shown in Figure 4. The CytoHubba plug-in in Cytoscape3.7.2 software was used to screen the 10 core genes, as shown in Figure 5.

### 3.5. GO Functional Enrichment Analysis and KEGG Pathway Enrichment Analysis

GO function enrichment analysis and KEGG pathway enrichment analysis were carried out by R software and Bioconductor database installation packages such as clusterProfiler and enrichplot. 1939 GO enrichment results were obtained (*P* < 0.05）, among which 1731 items of biological processes (BP) were closely related to the reactions of metal ions, blood circulation, reactive oxygen species, and oxidative stress, lipopolysaccharide, steroids, and bacterial origin molecules. The 141 items of molecular function (MF) are mainly related to protein phosphatase binding, nuclear receptor activity, and steroid receptor activity, transcription factor activity, cytokine activity, and receptor binding, NO synthase regulator activity, etc. 67 results of cell composition (CC) are mainly related to membrane microdomain, receptor complex, components, and inherent components of synaptic membrane and vesicle cavity, as shown in Figure 6.

In order to comprehensively study the role of JCWD in the prevention and treatment of VM, 156 pathways were screened by KEGG pathway enrichment analysis. It involves PI3K-Akt signal pathway, AGE-RAGE signal pathway, MAPK signal pathway, HIF-1 signal pathway, IL-17 signal pathway in diabetic complications, and signal pathways closely related to fluid shear stress and atherosclerosis, endocrine resistance, endometrial cancer, prostate cancer, etc., which mainly play an important role in inhibiting inflammatory reaction, hormone, and endocrine regulation. 20 pathways were selected for visualization, and the diagram is shown in Figure 7. In order to explore the role of JCWD in the signal pathway, a gene target-signal pathway network is constructed to identify the interaction between protein targets and signal pathways.  Figure 8 shows a target and pathway network composed of 55 target genes and 20 key pathways. The results of network analysis show that there are 17 targets whose values are greater than the average value of 8.67, which may appear in multiple pathways. Nine pathways had degrees greater than 2 times the mean degrees, which may also be regulated by multiple targets. In addition, there are synergies between the pathways.

### 3.6. Molecular Docking between Active Ingredients and Potential Targets

It is generally believed that the lower the binding energy of the molecular docking process, the better the affinity between the receptor and the ligand. Molecular docking results showed that the molecular docking affinity of quercetin, luteolin, kaempferol, tanshinone Iia, wogonin, naringenin, nobiletin, dihydrotanshinlactone, beta-sitosterol, and salviolone with core target proteins IL6, PTGS2, MAPK1, MAPK3, and CGRP1 were all less than −5.0 kcal/mol, and the results are shown in Table 3 and the docking results of the interaction between target proteins and the active components with the strongest binding activity, as shown in Figure 9.

## 4. Discussion

According to the universally recognized pathogenesis of VM, namely, the trigeminal neurovascular reflex theory, VM can be considered as a proinflammatory disease. It has been found that there is a close connection between the nervous system and the immune system, and inhibiting the expression level of inflammatory factors can reduce the symptoms of VM or the occurrence of VM [13].

Modern pharmacological studies have shown that Wendan decoction has the effects of anti-inflammation and regulating immune function [14]. Lin Huangguo et al. [15] found that Wendan decoction could reduce the levels of NF-*κ*B, TNF-*α*, and IL-6 in metabolic syndrome rats, indicating that Wendan decoction could inhibit the expression of inflammatory factors. Liu et al. [16] proved that Huanglian Wendan decoction could inhibit inflammatory reaction and reduce the levels of serum TNF-*α* and IL-6 in rats with metabolic syndrome. The research of Yu et al. [17] shows that Wendan decoction can effectively regulate the expression of TNF-*α*, IL-6, IL-17, and IL-22 and other related inflammatory cytokines in obese rats and improve the state of inflammatory reaction in obese rats. Dou et al. [18] found through experiments that modified Huanglian Wendan decoction could significantly improve the impairment of learning and memory and the pathological changes of hippocampus in rats with vascular dementia, reduce the expression of TNF-*α* and COX-2 in hippocampus, and play an inhibitory role in inflammatory response. Liu et al. [19] found that, in a certain glutamic acid environment, the drug-containing serum prepared with different doses of Wendan decoction could increase the survival rate of primary astrocytes P38MAPK extracted from the cerebral cortex of SD rats and upregulate the expression of P38MAPK phosphorylation and nonphosphorylation.

From the point of view of the active components of the drug, quercetin can exert its anti-inflammatory effect by inhibiting the production of IL-6, TNF-*α* and VEGF [20]. In addition, quercetin can exert its anti-inflammatory effect by inhibiting NF-*κ*B and MAPK signal pathways [21]. Kaempferol is a flavanol compound, which has many pharmacological effects, such as antioxidation and anti-inflammation. It can regulate the levels of NO and NOS and protect endothelial cells from oxidative damage by inhibiting the degradation of NO [22]. Luteolin mainly acts on transcription factors such as Src in the nuclear transcription factor-*κ*B (NF-*κ*B) pathway, MAPK in the activator protein-1 pathway, and cytokine signal inhibitors in the signal transduction and transcriptional activator 3 pathway, regulating inflammatory mediators and playing an anti-inflammatory role. Luteolin can inhibit all proinflammatory cytokines, such as interleukin-1*β*, IL-2, IL-6, IL-8, IL-12, IL-17, TNF-*α*, interferon-*β*(IFN-*β*), and granulocyte-macrophage colony stimulating factor and upregulate anti-inflammatory cytokine IL-10 [23]. Wogonin can inhibit the activation of both MAPK pathway and NF-*κ*B pathway, inhibit the expression of inducible nitric oxide synthase (iNOS), cyclooxygenase-2 (COX-2), TNF-*α*, IL-1*β* and IL-6, and reduce the inflammatory response of spinal dorsal root neurons induced by lipopolysaccharide [24,25]. Tanshinone IIA can inhibit the degradation of I*κ*B-*α* and the activation of NF-*κ*B induced by LPS by inhibiting the activation of NIK-IKK and MAPKs (p38, ERK1/2, JNK) signal pathways, so as to exert its anti-inflammatory activity [26].

Protein-protein interaction (PPI) network was used to screen out 10 core genes by Matthews correlation coefficient (MCC) algorithm. They are VEGFA (vascular endothelial growth factor A), MAPK3 (mitogen-activated protein kinase 3), MAPK1 (mitogen-activated protein kinase 1), EGF (epidermal growth factor), EGFR (epidermal growth factor receptor), IL-6 (interleukin-6), PTGS2 (prostaglandin endoperoxide synthase 2), STAT3 (signal transducer and activator of transcription 3), MMP9 (matrix metalloproteinase 9), and MMP2 (matrix metalloproteinase 2). Vascular endothelial growth factor (VEGF) has heparin active growth factor, which can play a role in vascular endothelial cells to cause the division and proliferation of vascular endothelial cells, thus forming new blood vessels and improving vascular permeability. The main causes of migraine include vasodilation and protein exudation. In the onset stage of migraine, patients' serum VEGF level is abnormally elevated, blood vessels dilate, and their permeability increases, eventually leading to extravasation of plasma protein [27]. Epidermal growth factor receptor (EGFR), widely expressed in the brain and aggregate distribution, is a functional receptor tyrosine kinase and, combined with neural regulatory proteins, can be changed after the epidermal growth factor receptor protein conformation, make its form dimers, and activate the downstream phosphatidyl inositol kinase/protein kinase B signaling pathway, which mediated inflammatory response [28]. MAPK is a class of intracellular serine/threonine protein kinases, an important signaling system that mediates extracellular signals to intracellular responses, and plays a key role in cell proliferation, apoptosis, inflammation, immunity, and angiogenesis [29]. Studies have observed changes in serum MMP9 levels in patients with migraine in different periods and subtypes and found that serum MMP9 was upregulated during the onset of migraine, which may be one of the potential related mechanisms of migraine [30]. IL-6 is a multipotent cytokine with a wide range of functions; it can regulate the growth and differentiation of many kinds of cells, regulate immune response, acute phase response and hematopoiesis, and play an important role in anti-infective immune response. PTGS2, also known as cyclooxygenase-2 (COX-2), is an enzyme that converts arachidonic acid into prostaglandins. It is overexpressed in response to mechanical, chemical, and physical stimuli and plays a key role in the promotion and development of inflammatory response [31,32]. Some studies have shown that COX-2 is involved in the pathogenesis of migraine, and the presence of aura has no effect on the level of serum COX-2, and some studies have suggested that exercise may improve the symptoms of vestibular migraine patients by inhibiting the COX-2 proinflammatory pathway and reducing the levels of TNF-*α*, IL-2, IL-6, and other proinflammatory factors [13].

Through the analysis of KEGG pathway, it is found that MAPK signal pathway, HIF-1 signal pathway, and IL-17 signal pathway are the main treatment pathways, which play a synergistic anti-inflammatory effect. MAPK signaling cascades include three different regulatory pathways: extracellular signal-regulated kinase (ERK1/2), c-jun N-terminal kinase (JNK) and p38 protein (P38), which are responsible for mitosis, proliferation, differentiation, and survival of cells during development [33], as well as neuronal plasticity and inflammation in adults [34]; in addition, these pathways contribute to the onset and maintenance of inflammation and pain [35]. In vitro studies have found that MAPK pathway can be involved in the upregulation of calcitonin gene-related peptide (CGRP) expression in rat trigeminal ganglion (TG) organ culture [36], and the release of CGRP and other neuropeptides is closely related to meningeal vascular inflammation and migraine symptoms. In addition, the transcription of COX-2 ′s PTGS2 gene is associated with multiple intracellular signals that come together to activate mitogen-activated protein kinase (MAPK) [37]. Based on the above discussion, we speculate that the possible mechanism of JCWD in the treatment of VM is shown in Figure 10.

## 5. Conclusion

In this study, the active components of JCWD and the potential targets and key pathways acting on vestibular migraine were predicted by the method of network pharmacology, which once again confirmed the process of multicomponent, multitarget, and multipathway treatment of diseases with traditional Chinese medicine compound prescription. The active components such as quercetin, kaempferol, luteolin, wogonin, and tanshinone II as in Jiawei Chaiqin Wendan decoction may regulate the levels of inflammatory factors and neurotransmitters (such as CGRP) by acting on IL6, MAPK3, MAPK1, PTGS2, and other targets, thus playing a role in the treatment of vestibular migraine. Due to the limitations of the database and the software itself, the above results need to be further verified by experiments.

## Figures and Tables

**Figure 1:** Venn diagram of the intersection target of JCWD and VM.

**Figure 2:** JCWD “drug-active compound-Gene Target” network diagram (where dark green represents the name of TCM, light green represents active ingredients, pink substitutes gene targets, and red color represents the name of the disease).

**Figure 3:** Protein-protein interaction network.

**Figure 4:** Degree ranking of top 20 target proteins.

**Figure 5:** Core genes of JCWD potential therapeutic targets.

**Figure 6:** GO enrichment analysis of 85 target genes. (a) Biological process enrichment analysis. (b) Cellular component enrichment analysis. (c) Molecular function enrichment analysis.

**Figure 7:** KEGG enrichment analysis of 85 target genes. (a) Barplot of KEGG analysis. (b) Dotplot of KEGG analysis: the size of dots indicates the number of target genes; the different color of dots indicates different *P* value ranges.

**Figure 8:** Targets-pathway network (the size of the icon represents the size of the degree value, the green rectangle represents the target gene, and the blue arrow represents the pathway.).

**Figure 9:** The molecular docking results of the interaction of active ingredients with the protein. (a) Binding pattern between IL-6 and dihydrotanshinlactone. (b) Binding pattern between PTGS2 and luteolin. (c) Binding pattern between MAPK1 and salviolone. (d) Binding pattern between MAPK3 and dihydrotanshinlactone. (e) Binding pattern between CGRP1 and quercetin.

**Figure 10:** Possible mechanism of JCWD for VM.

**Table 1:** Basic information of some active components of JCWD.

TCM	MOL ID	Molecule name	OB (%)	DL
Radix bupleuri	MOL002776	Baicalin	40.12	0.75
Radix bupleuri	MOL000449	Stigmasterol	43.83	0.76
Radix bupleuri	MOL000354	Isorhamnetin	49.6	0.31
Radix bupleuri	MOL000422	kaempferol	41.88	0.24
Radix scutellariae	MOL001689	Acacetin	34.97	0.24
Radix scutellariae	MOL000173	Wogonin	30.68	0.23
Radix scutellariae	MOL002714	Baicalein	33.52	0.21
Radix scutellariae	MOL002910	Carthamidin	41.15	0.24
Radix scutellariae	MOL002914	Eriodyctiol (flavanone)	41.35	0.24
Pinellia tuber	MOL002776	Baicalin	40.12	0.75
Pinellia tuber	MOL000358	Beta-sitosterol	36.91	0.75
Pinellia tuber	MOL000449	Stigmasterol	43.83	0.76
Pinellia tuber	MOL005030	Gondoic acid	30.7	0.2
Dried tangerine peel	MOL000359	Sitosterol	36.91	0.75
Dried tangerine peel	MOL004328	Naringenin	59.29	0.21
Dried tangerine peel	MOL005815	Citromitin	86.9	0.51
Dried tangerine peel	MOL005828	Nobiletin	61.67	0.52
Poria cocos	MOL000275	Trametenolic acid	38.71	0.8
Poria cocos	MOL000279	Cerevisterol	37.96	0.77
Poria cocos	MOL000283	Ergosterol peroxide	40.36	0.81
Poria cocos	MOL000289	Pachymic acid	33.63	0.81
Radix paeoniae alba	MOL001928	Albiflorin_qt	66.64	0.33
Radix paeoniae alba	MOL001930	Benzoyl paeoniflorin	31.27	0.75
Radix paeoniae alba	MOL000358	Beta-sitosterol	36.91	0.75
Radix paeoniae alba	MOL000359	Sitosterol	36.91	0.75
Fructus aurantii immaturus	MOL013276	Poncirin	36.55	0.74
Fructus aurantii immaturus	MOL013277	Isosinensetin	51.15	0.44
Fructus aurantii immaturus	MOL013279	5,7,4′-Trimethylapigenin	39.83	0.3
Fructus aurantii immaturus	MOL013428	Isosakuranetin-7-rutinoside	41.24	0.72
Fructus aurantii immaturus	MOL013430	Prangenin	43.6	0.29
Salvia miltiorrhiza	MOL001659	Poriferasterol	43.83	0.76
Salvia miltiorrhiza	MOL001771	Poriferast-5-en-3beta-ol	36.91	0.75
Salvia miltiorrhiza	MOL001942	Isoimperatorin	45.46	0.23
Salvia miltiorrhiza	MOL002651	Dehydrotanshinone II A	43.76	0.4
Angelica sinensis	MOL000358	Beta-sitosterol	36.91	0.75
Angelica sinensis	MOL000449	Stigmasterol	43.83	0.76
Uncariae ramulus cumuncis	MOL000358	Beta-sitosterol	36.91	0.75
Uncariae ramulus cumuncis	MOL000073	Ent-epicatechin	48.96	0.24
Uncariae ramulus cumuncis	MOL008457	Tetrahydroalstonine	32.42	0.81
Uncariae ramulus cumuncis	MOL008458	Angustidine	51.85	0.66

**Table 2:** Top 10 active ingredients by degree value.

MolID	Molecule name	Degree	Source
MOL000098	Quercetin	53	Radix bupleuri, uncariae ramulus cumuncis
MOL000006	Luteolin	21	Salvia miltiorrhiza, fructus aurantii immaturus
MOL000422	Kaempferol	19	Radix bupleuri, uncariae ramulus cumuncis, radix paeoniae alba
MOL007154	Tanshinone iia	16	Salvia miltiorrhiza
MOL000173	Wogonin	16	Radix scutellariae
MOL004328	Naringenin	13	Dried tangerine peel, fructus aurantii immaturus
MOL005828	Nobiletin	13	Fructus aurantii immaturus, dried tangerine peel
MOL007100	Dihydrotanshinlactone	13	Salvia miltiorrhiza
MOL000358	Beta-sitosterol	12	Radix paeoniae alba, pinellia tuber, radix scutellariae, angelica sinensis, uncariae ramulus cumuncis
MOL007145	Salviolone	12	Salvia miltiorrhiza

**Table 3:** The binding free energy of 10 small molecules with top 5 genes.

Molecule name	Affinity (kcal/mol)				
	IL6	PTGS2	MAPK1	MAPK3	CGRP
Beta-sitosterol	−5.9	−9.2	−7.5	−8.7	−6.7
Dihydrotanshinlactone	−7.8	−9.5	−8.9	−10.8	−8.2
Kaempferol	−7.6	−9.2	−7.7	−9.3	−9.0
Luteolin	−7.5	−10.0	−8.1	−9.4	−8.8
Naringenin	−7.2	−9.3	−8.0	−9.3	−8.5
Nobiletin	−6.2	−8.7	−6.9	−8.5	−7.9
Quercetin	−7.7	−9.6	−7.5	−9.3	−9.2
Salviolone	−7.2	−8.6	−9.1	−10.6	−7.7
Tanshinone iia	−7.6	−9.9	−8.6	−11.5	−7.9
Wogonin	−7.1	−9.4	−7.7	−9.3	−7.4

## Data Availability

The datasets used and/or analyzed during the current study are available from the corresponding author on reasonable request.
